This article has been retracted.

# Clinical Comparative Study of Intravitreal Injection of Triamcinolone Acetonide and Aflibercept in the Treatment of Diabetic Retinopathy Cystoid Macular Edema

**DOI:** 10.1155/2022/1348855

**Published:** 2022-05-18

**Authors:** Yanxia Zhu, Jun Li, Songping Yu, Bangxun Mao, Jia Ying

**Affiliations:** Department of Ophthalmology, Lishui Municipal Central Hospital, Lishui, Zhejiang 323000, China

## Abstract

*Objective* To compare the curative effect of intravitreal injection of triamcinolone acetonide and aflibercept on diabetic retinopathy (DR) cystoid macular edema. *Methods* A total of 102 patients with DR cystoid macular edema admitted to the hospital were enrolled between July 2018 and July 2021. According to random number table method, they were divided into the control group (intravitreal injection of triamcinolone acetonide) and the observation group (intravitreal injection of aflibercept), 51 cases in each group. All were followed up for half a year. The clinical curative effect, visual acuity, central subfield macular thickness (CSMT), macular volume, scores of quality of life, and levels of cytokines in aqueous humor (vascular endothelial growth factor (VEGF), monocyte chemoattractant protein-1 (MCP-1), human angiopoietin-like protein 4 (ANGPTL4)] at different time points (before and at 6 months after surgery) were compared between the two groups. The times of drugs injection and occurrence of adverse reactions in both groups were statistically analyzed. *Results* The total effective rate in observation group was higher than that in the control group (96.08% *vs* 82.35%) (*P* < 0.05). After 6 months of treatment, visual acuity was improved, and CSMT and macular volume were decreased in both groups. Also, the above changes were more significant in the observation group than those in the control group (*P* < 0.05). After 6 months of treatment, levels of cytokines in aqueous humor were decreased in both groups. The levels of VEGF, MCP-1, and ANGPTL4 in observation group were lower than those in the control group (*P* < 0.05). After 6 months of treatment, quality of life scores in observation group were higher than those in the control group (*P* < 0.05). In the follow-up period, average times of drugs injection in the observation group were more than those in the control group, and the incidence of adverse reactions was lower than that in control group (5.88% *vs* 21.57%) (*P* < 0.05). *Conclusion* The curative effect of intravitreal injection of both triamcinolone acetonide and aflibercept is good on DR cystoid macular edema. The curative effect of aflibercept is better, which can improve visual acuity and quality of life, and regulate cytokines in aqueous humor, with high safety. However, aflibercept has a high price, and further research is needed to determine whether its price can be matched with clinical benefits. In clinic, medication plan should be selected according to the actual situation.

## 1. Introduction

As a more serious ophthalmic complication of diabetes, diabetic retinopathy (DR) not only causes vision loss but even leads to blindness [1]. Cystoid macular edema is the leading cause of vision loss in DR patients [2]. With the increase of diabetic patients, the incidence of cystoid macular edema is also increased. In the past, the treatment of cystoid macular edema was laser grid photocoagulation or conservative drug treatment. However, the limitation of photocoagulation was to delay the progression of the disease, but it could not effectively improve vision. Therefore, it is imperative to explore new treatment methods for DR. There are foreign reports that vascular endothelial growth factor (VEGF) plays a key role in the pathogenesis of macular edema [3], it can stimulate the formation of new blood vessels and is expressed in the vitreous nucleus preretinal new blood vessels. Triamcinolone acetonide is a type of glucocorticoid, and aflibercept is an anti-VEGF drug that has been put into clinical use in recent years. The former has long-lasting effect and low price but leads to many complications [4]; the latter has good effect and less side effects, but it is expensive [5]. At present, the relevant reports on the treatment of DR cystic macular edema by these two methods are immature. In order to observe the exact curative effect, this study compared the effect of intravitreal injection of triamcinolone acetonide and aflibercept in the treatment of DR cystic macular edema.

## 2. Materials and Methods

### 2.1. Clinical Data

102 patients with DR cystic macular edema received in our hospital from July 2018 to July 2021 were selected and randomly divided into the control group and the observation group with 51 cases each group by the digital table method. The observation group included 31 males and 20 females, 53.82 ± 8.08 years old, and their duration of diabetes mellitus was 2.76 ± 0.95 years. The control group included 29 males and 22 females, 54.49 ± 9.17 years old, and their duration of diabetes mellitus was 2.86 ± 0.89 years. We compared the general data between the two groups, and the difference was not statistically significant (*P* > 0.05). This study complied with the relevant principles of the Declaration of Helsinki. The inclusion criteria are as follows: (1) meet the latest clinical diagnostic criteria for diabetes [6]; DR was diagnosed by fundus fluorescein angiography (FFA) and optical coherence tomography (OCT) and accompanied by cystic macular edema (cystic macular edema criteria [7]: foveal 500 mm retinal thickening, flattening, or hard exudation); (2) unilateral disease; (3) the family members of the patients were informed about the research and signed the consent form. The exclusion criteria are as follows: (1) other ocular diseases such as glaucoma and retinal detachment; (2) malignant tumors; (3) pregnancy or pregnant women; (4) have a history of eye surgery; (5) allergic to the study drug; (6) unable to cooperate with the examination or reexamination; (7) withdrawal from the treatment halfway.

### 2.2. Methods

The control group was treated with triamcinolone acetonide (1 ml/40 mg, Kunming Jida Pharmaceutical, National Medicine Permission Number H53021604), and the observation group was treated with aflibercept (1 ml/40 mg, Bayer, Germany, S20180010). Levofloxacin eye drops (5 ml/24.4 mg, Japan Santen Pharmaceutical Co., Ltd., National Medicine Permission Number J20150106) were used 3 days before operation, 4 times a day, washed the lacrimal duct half an hour before the operation, instilled eye drops, and in sterile operating room for operation, the patients were placed in a supine position to soothe the patients' emotions. After topical anesthesia, the eyes were sterilized, needled at the 4 mm pars plana of the corneal limbus, and 0.05 mL of aflibercept or triamcinolone acetonide was extracted to confirm that the needle was inserted into the vitreous cavity. Then, injected slowly, applied antibiotics to the conjunctival sac after withdrawing the needle, bandaged the eyes, and used eye drops for 1 week. All patients were followed up once a month after operation. According to the patient's condition, whether to supplement injection was decided. The follow-up lasted for six months.

### 2.3. Observation Indicators

(1) The two groups of patients underwent OCT examination 6 months before and after treatment, using frequency domain OCT (CirrusOCT, 6.0) produced by CarlZeiss Company, and 5-line high-definition scanning of the macular area. The visual acuity level, central subfield macular thickness (CSMT), and macular volume of the groups of patients before and after surgery were measured. (2) The anterior chamber of the corneal limbus of the patients was punctured 6 months before and after treatment, extracted 0.1 ml of aqueous humor, stored it at a low temperature immediately after collection, sent it for inspection, and used an immunoassay plate (Bole, USA), referring to the previous literature [8] to detect the level of VEGF and the mass concentration of monocyte chemoattractant protein-1 (MCP-1) and angiopoietin-like protein 4 (ANGPTL4). (3) The retinopathy quality of life scale [9] was used to evaluate the two groups of patients, which were divided into visual function, physical function, social activity, mental and psychological function, etc. The score was 0–200. The higher the score is, the better the quality of life will be. (4) During the follow-up, FFA was performed every time the patients were reexamined to check the occurrence of complications such as elevated intraocular pressure, cataract, and endophthalmitis.

### 2.4. Clinical Efficacy

The relevant literature [10] was referred to evaluate the efficacy of the two methods. Effectual: the symptoms of fundus oozing were significantly improved, and the visual acuity level improved by more than 2 lines on the visual chart; effective: the symptoms of fundus oozing were improved, and the visual acuity level improved 1–2 lines of improvement; invalid: there was no improvement or even worsening of fundus oozing symptoms, and no improvement in visual acuity.

### 2.5. Statistical Methods

The IBM SPSS Statistics 24.0 software was used to process the data in this study. The age, course of disease, visual acuity, CSMT and macular volume, aqueous cytokine levels, and quality of life scores of the two groups of patients were expressed as (*x* ± *s*). The *t*-test was used for comparison between groups; the clinical efficacy and adverse reactions of patients were expressed as rate (%); *χ*^*2*^ test was used between groups; and *P* > 0.05 was considered statistically significant.

## 3. Results

### 3.1. Comparison of Clinical Efficacy between the Two Groups

The results showed that the total effective rate of the observation group was 96.08%, which was higher than 82.35% of the control group (*P* > 0.05), as shown in Figure 1.

### 3.2. Comparison of Visual Acuity Levels between Two Groups of Patients at Different Times

The results showed that there was no significant difference in visual acuity level, CSMT value, and macular volume between the two groups before treatment (*P* > 0.05); after 6 months of treatment, the visual acuity level in both groups increased, CSMT value and macular volume decreased, and the changes in the observation group were more obvious (*P* > 0.05), as shown in Figures 2,3 and 4.

### 3.3. Comparison of VEGF, MCP-1, and ANGPTL4 Levels between the Two Groups of Patients

The results showed that there was no significant difference in the levels of VEGF, MCP-1, and ANGPTL4 between the two groups before treatment (*P* < 0.05). After 6 months of treatment, the levels of cytokines in the aqueous humor of the two groups were decreased, among which VEGF, MCP-1, and ANGPTL4 in the observation group were lower than those in the control group (*P* < 0.05), as shown in Figures 5, 6, and 7.

### 3.4. Comparison of Quality of Life Scores between the Two Groups of Patients

The results showed that there was no significant difference in the quality of life scores between the two groups before treatment (*P* < 0.05). After 6 months of treatment, the visual function, physical function, social activity, and mental and psychological quality of life scores of the observation group were higher than those of the control group (*P* < 0.05), as shown in Figures 8, 9, 10, and 11.

### 3.5. Comparison of Treatment-Related Indicators between the Two Groups of Patients

The results showed that in the follow-up period, the average number of injections in the observation group was more than that in the control group, and the incidence of adverse reactions was 5.88%, which was lower than 21.57% in the control group (*P* < 0.05), as shown in Figures 12 and 13.

## 4. Discussion

Macular cystic edema is the main cause of visual impairment of DR patients. After retinopathy in DR patients, ischemia and hypoxia occur, vascular permeability is enhanced, and the retinal barrier is damaged [11], which can easily lead to hard infiltration in the macular region of patients and edema occurs. Clinical treatment options include photocoagulation and intravitreal injection of drugs. The former may cause complications such as vision loss or visual field defect, while the latter injection of drugs such as glucocorticoid triamcinolone acetonide has certain curative effects, but it also has many adverse reactions. Aflibercept has been used well in recent years, and comparative studies with ranibizumab are more common [12, 13], while the comparative analysis of efficacy with triamcinolone acetonide is immature. Based on this background, the purpose of this study was to compare and analyze the efficacy of the two in the treatment of cystic macular edema, in order to contribute reasonable suggestions for the clinical treatment of DR patients.

An earlier foreign report indicated that [14] aflibercept, ranibizumab, or triamcinolone acetonide could effectively improve macular edema, while the intensity of the flare in the anterior part of patients eyes were only reduced when triamcinolone acetonide was treated. The results of this study showed that the effective rate of the observation group was higher than that of the control group, suggesting that the efficacy of intravitreal injection of aflibercept in the treatment of DR cystoid macular edema was significantly better than that of triamcinolone acetonide injection. Studies [15] have suggested that the efficacy of afenib in the treatment of DR is superior to that of ranibizumab, and the current comparative study with triamcinolone acetonide is rare, which needs to be confirmed by subsequent large sample size.

In addition, the results of this study found that the visual acuity level of the observation group was higher than that of the control group at 6 months after treatment, and the CSMT value and macular volume of the observation group were lower than those of the control group. This result indicates that intravitreal injection of aflibercept in the treatment of DR cystoid macular edema can effectively improve the visual acuity of patients, reduce macular volume and improve CSMT value. Glassman et al. [16] reported a similar view.

MCP-1 is a member of the chemokine CC family. As a proinflammatory factor, it can cause chemotaxis and activate monocytes and T lymphocytes. It has also been reported to be an effective indicator to reflect retinal inflammatory responses [17]. ANGPTL is cDNA amplified and cloned by foreign scientists in 1999. ANGPTL4 is mainly expressed in the liver and plays a key role in inflammation, angiogenesis, and tumors. Recent studies have shown that ANGPTL4 is a therapeutic target for retinopathy of DR patients [18]. At the same time, this study also found that the levels of VEGF, MCP-1, and ANGPTL4 in the two groups decreased after treatment, and the levels of VEGF, MCP-1, and ANGPTL4 in the observation group were lower than those in the control group, suggesting that intravitreal injection of aflibercept in the treatment of DR with macular edema can improve the cytokine levels in the aqueous humor. Recent foreign reports [19] also support this view. The reason may be that aflibercept contains an important domain of VEGF, which can bind to the receptor of the latter and block the downstream signaling pathway, thereby inhibiting VEGF-mediated chemotaxis of inflammatory cells and reducing the levels of VEGF, MCP-1, and ANGPTL4. In addition, the results of the study found that the quality of life scores in the observation group were significantly improved compared with those in the control group, reflecting that intravitreal injection of aflibercept played a role in better improvement of the quality of life of patients with DR and macular edema.

Finally, this study found that the incidence of adverse reactions in the observation group was lower than that in the control group, suggesting that intravitreal injection of aflibercept in the treatment of DR cystoid macular edema is safe, which is consistent with what Monés et al. [20] has proposed. However, the average number of injections in the observation group was higher than that in the control group. In recent years, a meta-analysis of pharmacoeconomics has shown [21] that the cost of aflibercept is significantly higher than that of ranibizumab and laser photocoagulation. Considered in connection with the conclusions of this study, multiple injections may bring a certain degree of medical burden to patients.

In conclusion, intravitreal injection of aflibercept and the treatment of cystoid macular edema in DR have definite curative effects and can improve visual acuity and quality of life, with good safety. However, because of the high price of aflibercept, multiple injections are often required to ensure the therapeutic effect, which will significantly increase the economic burden of patients. Whether the additional cost of this scheme is matched with the therapeutic benefit brought by this scheme still needs further investigation. In clinical use, treatment options should be selected according to the actual situation.

## Figures and Tables

**Figure 1:** Clinical efficacy of the two groups of patients. Compared with the control group, ^*∗*^*P* > 0.05.

**Figure 2:** Visual acuity levels of two groups of patients at different times. Compared with the same group before treatment, ^#^*P* < 0.05; compared with the control group, ^*∗*^*P* < 0.05.

**Figure 3:** CSMT values of two groups of patients at different times. Compared with the same group before treatment, ^#^*P* < 0.05; compared with the control group, ^*∗*^*P* < 0.05.

**Figure 4:** Macular volumes of two groups of patients at different times. Compared with the same group before treatment, ^#^*P* < 0.05; compared with the control group, ^*∗*^*P* < 0.05.

**Figure 5:** VEGF levels of two groups of patients at different times. Compared with the same group before treatment, ^#^*P* < 0.05; compared with the control group, ^*∗*^*P* < 0.05.

**Figure 6:** MCP-1 levels of two groups of patients at different times. Compared with the same group before treatment, ^#^*P* < 0.05; compared with the control group, ^*∗*^*P* < 0.05.

**Figure 7:** ANGPTL4 levels of two groups of patients at different times. Compared with the same group before treatment, ^#^*P* < 0.05; compared with the control group, ^*∗*^*P* < 0.05.

**Figure 8:** Visual function scores of the two groups of patients at different times. Compared with the same group before treatment, ^#^^*∗*^*P* < 0.05; compared with the control group, ^*∗*^*P* < 0.05.

**Figure 9:** Physical function scores of two groups of patients at different times. Compared with the same group before treatment, ^#^^*∗*^*P* < 0.05; compared with the control group, ^*∗*^*P* < 0.05.

**Figure 10:** The social activity scores of the two groups of patients at different times.Note: Compared with the same group before treatment, ^#^^*∗*^*P* < 0.05; compared with the control group, ^*∗*^*P* < 0.05.

**Figure 11:** The mental and psychological scores of the two groups of patients at different times.Note: Compared with the same group before treatment, ^#^^*∗*^*P* < 0.05; compared with the control group, ^*∗*^*P* < 0.05.

**Figure 12:** The average number of drug injections of the two groups of patients. Compared with the control group, ^*∗*^*P* < 0.05.

**Figure 13:** The occurrence of adverse reactions of the two groups of patients. Compared with the control group, ^*∗*^*P* < 0.05.

## Data Availability

The data presented in the study are included in the article. Further inquiries can be directed to the corresponding author.
